# Preoperative Lymphocyte-to-Monocyte Ratio Can Indicate the Outcomes in Repair of I-III Degree Injury of Lateral Ankle Ligament

**DOI:** 10.1155/2022/6234561

**Published:** 2022-04-19

**Authors:** Chengjie Yuan, Zhifeng Wang, Genrui Zhu, Chen Wang, Xin Ma, Xu Wang

**Affiliations:** Department of Orthopedics, Huashan Hospital, Fudan University, 12 Middle Wulumuqi Rd, Shanghai 200040, China

## Abstract

**Background:**

This study is aimed at exploring the prognostic value of preoperative lymphocyte-to-monocyte ratio (LMR), an index of systemic inflammation before operation, in ankle lateral ligament repair (ALLR).

**Methods:**

A total of 213 I-III degrees injuries of lateral ankle ligament patients received ALLR and were followed up for more than 2 years. Univariate and multivariable linear regression analysis was used to determine the relationship between preoperative LMR and postoperative recovery. The evaluations of postoperative recovery include American Orthopaedic Foot and Ankle Society (AOFAS) score, Karlsson-Peter ankle score (KPAS), Cumberland Ankle Instability Tool (CAIT) score, Visual Analog Scale (VAS) score, and range of motion (ROM). The prognostic value of preoperative LMR was measured by receiver operating characteristic (ROC) curve.

**Results:**

178 patients (178 ankles) were followed up successfully, with a follow-up of 2.82 ± 1.54 years. Overall, the mean AOFAS, KPAS, CAIT and VAS scores, and ankle varus angle were significantly improved at the final follow-up. Univariate and multiple linear regression analysis showed that preoperative LMR was the only independent factor associated with postoperative function, ROM, and pain. The preoperative LMR of patients with poor recovery was significantly lower than that of patients with good recovery. Based on the ROC analysis, the cutoff value of preoperative LMR was 3.824. The clinical outcomes of patients with preoperative LMR < 3.824 were significantly lower than that of patients with preoperative LMR ≥ 3.824. The corresponding specificity and sensitivity were 84.6% and 71.4%.

**Conclusion:**

The clinical outcomes of open or arthroscopic repair for ATFL injury are satisfactory. As a marker of systemic inflammation, preoperative LMR can be used as a prognostic indicator for ALLR.

## 1. Introduction

Lateral ankle sprain (LAS) is the most common ankle injury, of which 85% cumulative ankle anterior talofibular ligament (ATFL) [1]. And epidemiological studies reported that one ankle sprain occurs per 10000 people per day in the world. Waterman et al. reported that there were 3,140,132 ankle sprains from 2002 to 2006 (an average of 628,026 cases per year) in the 1.46 billion high-risk population and further estimated that the incidence of ankle sprains in the United States is 2.15 cases per 1,000 people per year [2]. Although most acute ankle sprains can be successfully treated by conservative methods, the epidemiological studies reported that 5-20% of ankle sprains will develop into chronic ankle instability (CAI) [3]. For these patients with CAI, operative repair of the ATFL is recommended. At present, the treatment techniques available for ATFL injury mainly include anatomical repair, such as Broström method, nonanatomical tenodesis, and anatomical reconstructions using allografts or autografts (peroneus brevis, gracilis, or semitendinosus) or synthetic grafts. Other nonanatomical techniques, such as the one described by Watson-Jones and Chrisman-Snook, involve the use of part of the patient's peroneus brevis tendon, with the double disadvantage of partial loss of function and nonisometry [4]. Usually, anatomical lateral ligament repair (ALLR) is the first choice [5]. Open or arthroscopic modified Broström-Gould procedure, considered as the gold standard for ALLR, has been widely used in the treatment of ATFL injury [6]. Based on previous clinical trials, ALLR usually leads to good anatomical and clinical results. However, in clinical practice, it is found that some patients still have inferior results, such as residual pain and limited range of motion (ROM), and these symptoms can last more than 2 years after operation.

Previous studies have examined the impact of many factors on the outcomes of ALLR. Demographic descriptive factors include age, gender, and BMI. Intraoperative factors included operative technique. The characteristics of ATFL injury include the grade of ligament injury, combined cartilage injury or impact, and the symptom duration. Thompson et al. found that age and ligament injury grade were independent factors of poor recovery, but they could not be regarded as a reference [7].

In addition to these factors, previous studies have reported that local inflammatory factors are also associated with poor prognosis after ALLR. It has been found that chronic synovitis in the anterolateral ankle, as well as increased leukocyte infiltration or interleukin levels, may mediate ankle pain and functional limitation. [8]. At the same time, the proinflammatory factors and chemokines induced by repeated mechanical stretch injury of ATFL are also related to the persistent pain after ALLR. Thomas et al. found that the polymorphisms of inflammatory factors in ankle, such as the increase of stromal cell-derived factor-1(SDF-1) and matrix metalloproteinase-13 (MMP-13), were associated with postoperative ankle dysfunction [9]. What is more, systemic inflammatory factors also have a role in the recovery process after ALLR. For patients with diabetes, hypertension, gout, and osteoporosis, the increase of systemic inflammation is a common feature, and the incidence of residual pain, feeling of instability, and limited ROM after ALLR is higher [10]. Therefore, evaluating the level of systemic inflammation before ALLR may help to predict the postoperative outcomes.

Clinically, C-reactive protein (CRP), erythrocyte sedimentation rate (ESR), and procalcitonin (PCT) are commonly used to evaluate the level of systemic inflammation [11]. However, whether CRP, ESR, or PCT are elevated in systemic inflammation-related diseases remains controversial. Harrison et al. think that ESR may be affected by many noninflammatory factors, and CRP is mainly caused by the response of hepatocytes to interleukin-6 (IL-6) [12, 13]. At the cellular level, as part of the immune system, lymphocytes and monocytes mediate inflammation and are also regulated by inflammation [14]. In recent years, an increasing amount of evidence shows that it is of comprehensive significance to use lymphocyte-to-monocyte ratio (LMR) to reflect the level of systemic inflammation. Kocak et al. [15] confirmed the relationship between LMR and diabetes, and Ye et al. [16] found that LMR is also related to osteoporosis, in which lower LMR represents a higher level of inflammation, promoting the occurrence and development of related diseases.

At present, the research on LMR affecting the outcomes of ALLR is limited, and the understanding of the independent predictors for ALLR is also limited. Considering the association between systemic inflammatory status and the outcomes of ALLR, we included a variety of factors, including preoperative demographic data, preoperative systemic inflammatory index LMR, intraoperative factors, and patient factors. We then evaluated the relationship between these preoperative and intraoperative factors and postoperatively clinical outcomes. Our hypothesis is that preoperative LMR can be an independent predictor of the outcome of ALLR.

## 2. Methods

ATFL injury patients who underwent open or arthroscopic ALLR from January 2014 to December 2018 were included. The inclusion criteria were as follows: (1) magnetic resonance imaging (MRI) and (or) B-ultrasound showed ATFL injury of ankle, (2) preoperative stress X-ray showed that the talus moved forward more than 10 mm, and the talus inclination was more than 5 degrees in varus stress test, and (3) at least 2 years of follow-up. The exclusion criteria were as follows: (1) any foot or ankle arthritis, (2) all types of ankle and (or) foot deformities, (3) history of ipsilateral ankle and (or) foot operation, (4) history of ipsilateral Achilles tendon injury, tendinopathy, and operation, (5) the ipsilateral ankle joint was injured or operated again after ALLR, (6) postoperative infection, (7) local steroids injection within 3 months before operation, (8) autoimmune diseases, and (9) cyst or tumor of foot and ankle. This study was approved by the institutional review committee of the hospital.

All procedures were performed by a senior surgeon (the corresponding author). All patients were given general anesthesia, and the stress radiographs were taken under anesthesia. All patients were in supine position, and the affected ankle was in neutral position. For open Broström-Gould procedure, 2-4 cm incision was made along the lower edge of lateral malleolus to expose the lower extensor retinaculum. After entering the joint, the torn end of ATFL was found. A 2.8 mm titanium anchor (Arthrex, Naples, FL) was single loaded at the fibular insertion of the ATFL. The ligament stump was sutured in the neutral position of the ankle. The lower extensor retinaculum was partially separated and sutured to the local capsule (Gould modified procedure). After suturing the wound, a cast was performed in the neutral position.

Total arthroscopy Broström-Gould procedure, the anterior medial entrance was made through an incision of 1 cm along the anterior tibialis tendon. Arthroscopic exploration was performed of the insertion of the ATFL. Under the arthroscopic control, a lateral incision of 1 cm was made above the fibula insertion of ATFL. Radiofrequency ablation was performed on the scar tissue. A 2.8 mm titanium anchor (Arthrex) was placed at the fibular insertion of ATFL. The anchor suture was introduced into the ligament stump with a guide wire, and the ligament stump was tightened when the ankle was in the neutral position. Then, the lower extensor retinaculum was sutured to the local capsule to strengthen. After suturing the wound, a cast was performed in a neutral position.

The short leg cast was removed within 4 weeks after operation, and nonweight bearing flexion and extension of the hip, knee, and ankle were encouraged. At 4-6 weeks after operation, patients began to walk in a boot. The rehabilitation strategies include ankle range of motion exercise and lower limb muscle strength exercise. The flexion and extension of the ankle were passively performed, and strengthening exercises of the whole lower extremity were started. Balance training and full weight-bearing training were performed 6-12 weeks after operation. We instructed the patient to use celecoxib for 1 week after operation.

The clinical independent variables were divided into 5 categories: (1) descriptive variables, including age, gender, BMI, and affected side; (2) the systemic inflammatory index LMR was defined as the ratio of lymphocyte count and monocyte count measured by blood routine 1 day before operation; (3) the characteristics of ATFL injury, including the duration from onset of symptom to operation, the grade of ligament injury, osteochondral lesions of the talus (OLT), trauma, and synovitis; (4) intraoperative factors, including operative technique (open or arthroscopic repair); (5) previous history, including hypertension, diabetes, gout, osteoporosis, history of nonsteroidal drugs, smoking, and drinking; and (6) preoperative functional score, pain score, and range of motion (ROM), including American Orthopaedic Foot and Ankle Society (AOFAS) score, Karlsson-Peterson ankle score (KPAS) score and Cumberland Ankle Instability Tool (CAIT) score, Visual Analog Scale (VAS) score, passive ankle plantarflexion, dorsiflexion, and varus and valgus angles.

Ankle function scores, VAS score, and ROM were assessed and collected by an experienced orthopedic specialist before surgery and at the last follow-up. The 3 ankle function scores included AOFAS score, KPAS score, and CAIT score. The VAS score is used to assess the level of pain before and after operation. ROM was measured by goniometer including passive ankle plantarflexion, dorsiflexion, and varus and valgus angles. Varus and valgus angles also indicate the stability of ankle. Poor postoperative recovery was defined as AOFAS score < 80 [17]. Postoperative ROM limitation was defined as ankle plantarflexion + dorsiflexion ≤ 30 degrees [18]. Residual pain was defined as postoperative VAS score > 3. At least 2 years after operation, 3.0T MRI with an 8-channel phase ankle coil was used to evaluate the continuity of ATFL. If the anterior drawer test (ADT) and talus tilt test were positive and the continuity of ATFL was lost, it was defined as postoperative retear. And all the examinations were completed by a same senior surgeon (corresponding author).

The analysis was performed with SPSS 21.0 software (SPSS Inc) and GraphPad Prism 7.0. Data were expressed as mean and standard deviation or the number of cases. First, to examine the improvement degree between pre- and postoperative clinical outcomes, the Student *t*-test or Mann–Whitney *U* test was conducted based on the test of normality and the Levene test for equality of variances. Chi-square test was used to detect the differences between binary variables. Ordinary least square (OLS) regression analysis was conducted to detect the association between preoperative clinical variables and postoperative outcome measures. And then collinearity analysis was used for testing the interaction between independent variables and controlling for candidate confounding. Finally, multivariable linear regression analysis was adopted when >1 factor was significantly associated with 1 postoperative outcome measures. The association strength was weak when the coefficient *B* < 0.4, moderate if 0.4 ≤ |*B*| < 0.7, and strong if 0.7 ≤ |*B*| < 1. In addition, receiver operating characteristic (ROC) curve and Youden index were used to determine the cutoff value. *P* < .05 was considered statistically significant. Essentially, the analysis of this study is exploratory in nature.

Since no previous study can be used to test the diagnostic value of LMR in the recovery of ALLR, the sample size cannot be calculated before patient registration. Therefore, based on the specificity and sensitivity we obtained, a post hoc calculation was launched with 15.0 software (NCSS Inc) instead. The type I error was set as.05, and the permissible error of 10% was set with regard to specificity and sensitivity.

## 3. Results

A total of 213 patients were included in this study, and 178 patients (83.57%) were successfully followed up for more than 2 years.  Table 1 shows the all clinical variables of all included patients, and preoperative values of the outcome measures (VAS, AOFAS, KPAS, CAIT, dorsiflexion, plantarflexion, varus, valgus) were also included as predictor variables. No infection or other complications occurred after the operation. As expected, patients improved in function, pain, and ROM postoperatively. The changes of passive dorsiflexion, plantarflexion, and valgus remained unremarkable (Table 2). At the last follow, 10 patients had retear based on MRI and physical examination (5.62%).

Next, the relationship between LMR and the postoperative outcomes were analyzed using the OLS regression analysis. And the specific data were shown in Table 3. An OLS regression analysis was also conducted between other descriptive information, preoperative, intraoperative factors, and postoperative outcomes (Table 4).

In order to further confirm whether LMR, gender, diabetes, and synovitis were independently associated to postoperative ankle function, ROM, and stability, collinearity analysis and multivariable linear regression analysis were conducted successively. The results of collinearity analysis indicated that there is no multicollinearity relationship between the four predictor variables (sex: VIF = 1.08, tolerance = 0.92; LMR: VIF = 1.15, tolerance = 0.87; synovitis: VIF = 1.08, tolerance = 0.92; diabetes: VIF = 1.11, tolerance = 0.90), which provided confidence in the next multivariable linear regression analysis. Eventually, the results of multivariable linear regression showed that only preoperative LMR was significantly associated with KPAS (*B* = 2.62, *P* < .001) (Table 5). In conclusion, preoperative LMR was the only independent factor during this follow-up period, which was associated with postoperative function (indicated by AOFAS score, KPAS, CAIT score), pain (indicated by VAS score), and ROM (indicated by dorsiflexion, plantarflexion, varus and valgus). In contrast, LMR did not show a significant association with postoperative retear.

The distribution of cases with either poor function, limited ROM, and pain or a combination was shown in Figure 1. Compared with the counterparts, the patients with poor function (4.41 ± 0.66 vs. 5.31 ± 1.62, *P* = .004), postoperative limited ROM (3.52 ± 0.94 vs. 4.88 ± 1.64, *P* = .027), and residual pain (4.16 ± 1.12 vs. 4.97 ± 1.43, *P* = .033) had significantly lower LMR, representing a high inflammation status (Figure 2).

Next, the ROC curve was calculated to determine the prognostic value of preoperative LMR on postoperative outcomes. The results showed the that area under curve (AUC) was 0.805, cut-off value was 3.824, and Youden index was 0.560. Sensitivity was 71.4% with a specificity of 84.6% (Figure 3). The post hoc sample size calculation shows that 85 cases were required to achieve the statistical significance of sensitivity, and 121 cases were required to achieve the statistical significance of specificity. Since 178 patients were included in this study, the diagnostic data obtained were reliable.

Based on cutoff value (LMR = 3.824), the patients were divided into groups, of which 62 patients had an LMR < 3.824. The pre- and postoperatively clinical measurements were shown in Table 6. For the 2 groups of patients classified by cutoff value (LMR = 3.824), the cutoff of AOFAS score and DF + PF angle were used to categorize patients again in each group. We found that the proportion of patients with AOFAS < 80 or DF + PF ≤ 30 degrees in patients with LMR < 3.824 was significantly higher than that of patients with LMR ≥ 3.824. Compared with patients with LMR ≥ 3.824, patients with LMR < 3.824 had a significantly higher risk of poor function and postoperatively limited ROM, with a risk ratio of 2.222 (95% CI, 1.233-4.005) and 2.432 (95% CI, 1.132-5.225), respectively (Figure 4).

## 4. Discussion

Based on the current study, for patients with ATFL injury without severe local comorbidities (such as ankle arthritis or deformity), a low LMR level, representing high systemic inflammatory status, was an independent factor associated with functional recovery, pain, and ROM after ALLR. The sensitivity and specificity of LMR were 71.40% and 84.60%, respectively. The risk of poor function in patients with LMR < 3.82 was 2.22 times higher, and the risk of limited ROM was 2.43 times higher at >2 years postoperatively.

Open or arthroscopic modified Broström-Gould procedure is a common operation in foot and ankle surgery. It usually has a satisfactory outcome for the ATFL injury, and patients usually return to their exercise level before injury 2 years postoperatively. Rocco et al. [19] reported that in a study with follow-up over 2 years, there was no significant difference in AOFAS score, KPAFS, and VAS score and total complication rate of open and arthroscopic ALLR. The total follow-up time was 25.9 months. The AOFAS score ranged from 70.90 to 95.33, KPAFS ranged from 73.50 to 93.41, and VAS score ranged from 1.2 to 2.1. In our cohort with degree I-III ATFL injury, patients were followed up for 2.82 ± 1.54 years with a mean AOFAS score of 85.02, KPAFS of 82.77, and VAS score of 1.78 postoperatively. Our postoperative outcomes suggested a similar recovery to those previous literatures on postoperative function, ROM, and pain. Maffulli et al. reported a study with follow-up of 8.7 years and found that 21.05% of the patients had poor postoperative function treated with modified Broström-Gould procedure [20]. Adam et al. analyzed the patients treated with modified Broström-Gould procedure with a follow up of 64 months [6]. However, the results suggested that 17% of the patients still experienced inferior functional outcomes (AOFAS < 80) in the last follow-up. Similarly, in our cohort, 35 patients had poor functional outcomes (19.66%) at 2.82 years after operation.

Regarding ROM reduction or limitation after ALLR, Ziaei Ziabari et al. suggested that the ROM of 16% patients after ALLR was smaller than that of the corresponding contralateral ankle [21]. They inferred that it is mainly due to too tight suture, local inflammation, and scar adhesion. The incidence of ROM reduction in our cohort was 12.92%, slightly lower than that reported in literatures. In addition to our emphasis on the improvement of operational techniques and postoperative rehabilitation, one possible reason is the definition of postoperative ROM limitation. In four studies included by Ziaei Ziabari et al., ROM limitation was defined as less ROM than the contralateral ankle postoperatively [21]. In this study, ROM limitation was defined as DF + PF < 30 degrees, which was adopted from studies published by Ozeki et al. [18]. Ozeki et al. found that during ankle movement, the tension of ATFL fiber was 0 N if plantarflexion ≤ 16 degrees, and the tension of PTFL and CFL fiber was 0 N if dorsiflexion ≤ 18 degrees. Therefore, when the ROM is less than this range (DF + PF < 34 degrees), it means the tension of lateral ligament complex of ankle increases during normal gait. At the same time, the value also meets the requirement of minimum plantarflexion and dorsiflexion (DF + PF = 30 degrees) for human to go up and down stairs normally. [22] Therefore, DF + PF < 30 degrees was determined as a definition of ROM limitation.

Ankle function and ROM have been thought to be linked to systemic conditions, such as the increase of SDF-1 and MMP-13 are related to poor ankle function [9]. Among other joints, studies focused on shoulder has made it clear that stiffness and loss of function are related to the systemic inflammation status, which reported that systemic inflammation has causal relationship with shoulder function, pain, and ROM [23, 24]. Ankle joint, as a joint with stability and flexibility, limited studies reported about the effects of systemic or local inflammation on its function and ROM. Among the factors related to the poor recovery after ALLR, many diseases are related to systemic inflammation, such as aging, diabetes, osteoporosis, and gout [25]. Therefore, systemic inflammation status may be valuable in predicting the outcome of ALLR postoperatively.

In recent years, the research on systemic inflammation has focused on the proportion of various kinds of leukocytes in blood, among which LMR has been suggested predictive role in many inflammatory statuses, such as cancer or diabetes and related complications [26, 27]. The lower LMR would indicate higher systemic inflammation and vice versa. In the current study, we found that LMR was the only factor independently associated to ankle function, ROM, stability, and pain after ALLR. In addition, the patients with poor function (AOFAS < 80) or postoperative stiffness (DF + PF ≤ 30 degrees) had lower mean preoperative LMR than that of good function (AOFAS ≥ 80) or ROM (DF + PF > 30 degrees). And in patients with LMR < 3.82, the proportion of patients with poor function (AOFAS < 80) or postoperative stiffness (DF + PF ≤ 30 degrees) was higher than that of patients with LMR ≥ 3.82. These results indicate that LMR has prognostic value for ankle function and ROM after ALLR.

The LMR of the population aged 30-39 ranged from 2.10 to 8.86, with an average of 5.48 [28]. The average age of patients in our cohort was 34.67 years, and the average LMR was 4.75. So far, a consensus on LMR threshold to indicate inflammatory status has not been reached [26]. The cutoff value (LMR = 3.82) obtained in this study was based on the regression analysis between the preoperative LMR and postoperative outcomes of 178 patients with ATFL injury accepted ALLR. Therefore, there is still a need for further studies with larger cohorts for verification.

Due to the biomechanical particularity of the coupling of ankle, many factors that would affect the recovery of ALLR have been clarified in previous literatures [29]. Traumatic ankle arthritis, subtalar arthritis, and injury of inferior tibiofibular syndesmosis, etc. are all the proven factors. Therefore, these patients were excluded from the current study cohort. However, the relationship between age, gender, duration of symptoms, grade of ligament injury, operational technique, OLT, and recovery after ALLR is still controversial. O'Connor et al. concluded that age, ligament injury grade, and weight-bearing status were only related to short-term postoperative recovery [30]. Akacha et al. supported that gender was a factor influencing the delay of short-term recovery after ALLR, but it was not related to the medium and long-term postoperative recovery [31]. Langner et al. suggested that severe ATFL injury was associated with longer postoperative recovery time [32]. Sun et al. found that there was no significant difference in postoperative outcomes (AOFAS, KPAFS, Talar tilt, ADT, complications) between open or arthroscopic ALLR [33]. In our cohort, the basic demographic characteristics, preoperative, and intraoperative factors (except for LMR) have not been found to be associated with postoperative recovery. In addition, imitated by factors included in this study, further studies could verify the effect of more other factors on postoperative recovery in a larger cohort.

In the current study, the relationship between some diseases (such as diabetes, synovitis) and postoperative recovery of ALLR remains debatable. We did not detect a relationship between diabetes or synovitis in multivariable linear regression analysis, which may be associated with fewer patients included in diabetes or synovitis in the current cohort. Considering that diabetes and synovitis are related to some outcomes postoperatively in univariate analysis, as well as different complications and treatments have different effects on the systemic inflammatory status, LMR could be recommended as an indicator of systemic inflammatory status instead of a certain physical disease to predict recovery.

Based on the large number of cases, this study first explored the prognostic value of LMR on the postoperative results of ALLR for ATFL injury. A variety of statistical methods were used to improve the reliability of the research results. Preoperative LMR can be used as a prognostic indicator for ALLR, which may help to reveal the relationship between preoperative systemic inflammation and postoperative lateral ankle ligament injury. This study is helpful for surgeons to judge the prognosis of patients with ankle instability by referring to LMR before operation, so as to carry out accurate treatment and rehabilitation exercise during and after operation, which is conducive to providing the curative effect of ALLR operation for ATFL injury and improving the quality of life of patients.

There are some limitations in this study. There are many joints in foot and ankle, and the biomechanical mechanism is very complex. The practicability of LMR cutoff value before operation needs more verification in other conditions. In addition, we only analyzed the relationship between LMR 1 day before operation and postoperative measurements. Continuous monitoring may be required, given that LMR may vary with age, medication, or other factors during follow-up. However, the prognostic value of a single preinterventional LMR for the prognosis of other various diseases has been proven before, making our finding credible. In addition, since there were no previous studies analyzed the relationship between LMR and postoperative recovery of ALLR, we were unable to calculate the sample size before patient registered; so, more studies with large sample were needed to test our findings. Finally, although we have customized a set of standard rehabilitation procedures after the patients were discharged, the degree of patient implementation is different, which may have a certain impact on the results. In the follow-up study, the variable of postoperative rehabilitation needs to be controlled more accurately, which would make the results more credible.

## 5. Conclusion

In general, the ALLR for ATFL injury in our center is satisfactory. However, the postoperative function, ROM, and pain results of some patients are still not ideal and associated to systemic inflammatory status. Preoperative LMR could be used as a systemic inflammatory marker to be predictive for outcomes after ALLR.

## Figures and Tables

**Figure 1:** Distribution of patients with American Orthopaedic Foot and Ankle Society (AOFAS) score < 80, dorsiflexion + plantarflexion (DF + PF) ≤ 30 degrees, Visual Analog Scale (VAS) score > 3, or combinations.

**Figure 2:** Difference of lymphocyte monocyte ratio between groups with (a) American Orthopaedic Foot and Ankle Society (AOFAS) score < 80 and ≥ 80, (b) Visual Analog Scale (VAS) score > 3 and ≤ 3, and (c) dorsiflexion + plantarflexion (DF + PF) ≤ 30 degrees and > 30 degrees.

**Figure 3:** Receiver operating characteristic (ROC) curve to determine the prognostic cutoff value of lymphocyte monocyte ratio (LMR) for poor outcomes defined as American Orthopaedic Foot and Ankle Society (AOFAS) score < 80.

**Figure 4:** The proportion of patients with (a) American Orthopaedic Foot and Ankle Society (AOFAS) score < 80 or (b) dorsiflexion + plantarflexion (DF + PF) ≤ 30 degrees when grouped by lymphocyte monocyte ratio (LMR).

**Table 1:** Basic preoperative and intraoperative characteristics of ATFL injury patients enrolled.

	Values
No. of ATFL injury patients (no. male)	178 (100)
No. of ankles (no. male)	178 (100)
No. of left side (no. right)	90 (88)
Age, y	34.67 ± 10.24 (range, 15 to 68)
Height, cm	170.15 ± 8.54 (range, 150 to 193)
Weight, kg	70.92 ± 12.98 (range, 45 to 98)
Body mass index, kg/m^2^	24.34 ± 3.11 (range, 18.03 to 30.99)
Follow-up, y	2.82 ± 1.54 (range, 2.16 to 6.41)
Lymphocyte count	30.53 ± 7.21
Monocyte count	6.82 ± 1.78
Lymphocyte monocyte ratio	4.75 ± 1.64 (range, 1.33 to 10.00)
Symptom duration, m	15.65 ± 18.96 (range, 1 to 96)
Patient factors	
AOFAS score	51.87 ± 15.73
KAPS score	40.57 ± 17.2
CAIT score	15.48 ± 4.50
VAS score	4.98 ± 1.64
Plantarflexion	44.33 ± 5.83
Dorsiflexion	24.63 ± 5.11
Varus	20.53 ± 2.91
Valgus angles	15.22 ± 3.18
Osteochondral lesions of the talus	61
Arthroscope procedure (no. open repair)	64 (114)
Trauma	77
Synovitis	50
Gout	4
Diabetic mellitus	19
Hypertension	28
Osteoporosis	3
Smoking	14
Alcoholism	9
Nonsteroidal anti-inflammatory drugs history within 3 months prior to surgery	36
Degree of ligament injury	
I	50
II	58
III	70

**Table 2:** The difference between preoperative and postoperative clinical measurements^a^.

Measurements	Preoperative	Postoperative	*T*	*P* value
American Orthopaedic Foot & Ankle Society score	51.87 ± 15.73	85.02 ± 9.55	-14.52	<0.001^∗∗^
Karlsson-Peterson ankle score	40.57 ± 17.2	82.77 ± 8.70	-19.30	<0.001^∗∗^
Cumberland Ankle Instability Tool score	15.48 ± 4.50	25.02 ± 2.82	-15.73	<0.001^∗∗^
Visual Analog Scale score	4.98 ± 1.64	1.78 ± 1.11	12.85	<0.001^∗∗^
Dorsiflexion, deg	24.63 ± 5.11	25.11 ± 3.69	-0.61	0.546
Plantarflexion, deg	44.33 ± 5.83	42.97 ± 3.61	1.47	0.132
Ankle varus deg	20.53 ± 2.91	19.12 ± 3.69	2.31	0.024^∗^
Ankle valgus, deg	15.22 ± 3.18	14.80 ± 3.15	0.75	0.455
Retear		10		

^a^Preoperative and postoperative values are showed as mean ± SD; ^∗^*P* < 0.05, ^∗∗^*P* < 0.001.

**Table 3:** Association between preoperative lymphocyte monocyte ratio and postoperative measurements.

Measurements	Regression coefficient (*R*)	*P* value
American Orthopaedic Foot & Ankle Society score	0.641	<.001^∗^
Karlsson-Peterson ankle score	0.526	<0.001^∗∗^
Cumberland Ankle Instability Tool score	0.627	<0.001^∗∗^
Visual Analog Scale score	-0.337	0.008^∗^
Dorsiflexion, deg	0.291	0.024^∗^
Plantarflexion, deg	0.324	0.011^∗^
Varus, deg	-0.395	0.002^∗^
Valgus, deg	-0.323	0.012^∗^
Retear	0.166	0.205

^∗^ *P* < 0.05, ^∗∗^*P* < 0.001.

**Table 4:** The *P* value of regression analysis between clinical variables and patient factors with postoperative outcomes^a^.

Factors	Outcomes								
	AOFAS	KPAS	VAS	CAIT	DF	PF	VAR	VAL	Retear
Age	0.923	0.727	0.681	0.874	0.928	0.938	0.740	0.863	0.608
Sex	0.183	0.045 (0.260)^∗^	0.787	0.186	0.871	0.085	0.157	0.285	0.562
Side	0.947	0.235	0.108	0.935	0.814	0.644	0.924	0.531	0.306
Body mass index	0.545	0.652	0.152	0.505	0.701	0.506	0.398	0.537	0.216
Symptom duration	0.809	0.358	0.281	0.970	0.834	0.896	0.809	0.682	0.676
Osteochondral lesions of the talus	0.912	0.582	0.476	0.751	0.222	0.532	0.222	0.271	0.332
Arthroscope procedure	0.753	0.681	0.768	0.729	0.627	0.719	0.735	0.144	0.281
Trauma	0.621	0.742	0.501	0.625	0.258	0.225	0.680	0.245	0.171
Synovitis	0.107	0.595	0.781	0.114	0.018 (-0.304)^∗^	0.231	0.038 (-0.268)^∗^	0.042 (-0.263)^∗^	0.281
Gout	0.184	0.501	0.890	0.190	0.307	0.751	0.208	0.227	0.649
Diabetic mellitus	0.112	0.044 (-0.262)^∗^	0.963	0.093	0.147	0.300	0.024 (-0.291)^∗^	0.240	0.351
Hypertension	0.274	0.681	0.916	0.300	0.464	0.813	0.592	0.658	0.103
Osteoporosis	0.324	0.976	0.766	0.348	0.603	0.641	0.573	0.876	0.810
Smoking	0.609	0.808	0.686	0.626	0.965	0.917	0.651	0.715	0.335
Alcoholism	0.325	0.732	0.777	0.455	0.630	0.194	0.484	0.093	0.601
Degree of ligament injury	0.096	0.114	0.445	0.121	0.010	0.130	0.028	0.418	0.824
NASAIDs	0.408	0.541	0.576	0.400	0.540	0.509	0.250	0.508	0.528

^a^AOFAS: American Orthopaedic Foot & Ankle Society score; KPAS: Karlsson-Peterson ankle score; CAIT: Cumberland Ankle Instability Tool score; VAS: Visual Analog Scale score; DF: dorsiflexion; PF: plantarflexion; VAR: varus; VAL: valgus. ^∗^The difference reached statistical significance (*P* < 0.05), with the specific regression coefficient given in parentheses.

**Table 5:** Multiple linear regression analysis between variables suspected to be related to recovery and affected postoperative measurements^a^.

Factors	Outcomes				
		KPAS	DF	VAR	VAL
Lymphocyte monocyte ratio	*β*	2.623	0.584	0.766	0.507
	*P*	<0.001^∗^	0.044^∗^	0.009^∗^	0.041^∗^
Sex	*β*	1.967	NA	NA	NA
	*P*	0.355	NA	NA	NA
Synovitis	*β*	NA	-1.475	-1.621	-1.315
	*P*	NA	0.122	0.085	0.106
Diabetic mellitus	*β*	-0.722	NA	-1.083	NA
	*P*	0.829	NA	0.482	NA

^a^KPAS: Karlsson-Peterson ankle score; DF: dorsiflexion; VAR: varus; VAL: valgus. ^∗^The association showed statistical significance (*P* < 0.05) with specific coefficient (*β*) marked.

**Table 6:** Comparison of pre- and postoperative measurements in patients with different preoperative lymphocyte monocyte ratios^a^.

	Patients with LMR < 3.824 (*n* = 62)			Patients with LMR ≥ 3.824 (*n* = 116)			Intergroup comparison	
	Preoperative	Postoperative	Intragroup comparison	Preoperative	Postoperative	Intragroup comparison	Preoperative difference	Postoperative difference
AOFAS	53.52 ± 10.01	80.86 ± 5.00	<.001^∗^	54.05 ± 15.4	87.26 ± 7.46	<.001^∗^	.888	.001^∗^
KPAS	40.19 ± 11.21	80.38 ± 4.42	<.001^∗^	40.90 ± 13.19	84.08 ± 5.77	<.001^∗^	.836	.013^∗^
CAIT	14.43 ± 4.59	24.71 ± 1.79	<.001^∗^	16.05 ± 4.40	26.26 ± 2.27	<.001^∗^	.185	.011^∗^
VAS	5.19 ± 1.36	2.29 ± 0.85	<.001^∗^	4.62 ± 1.31	1.51 ± 1.14	<.001^∗^	.115	.009^∗^
DF, deg	25.62 ± 4.67	23.81 ± 4.06	.186	24.10 ± 5.32	25.82 ± 3.32	.078	.277	.043^∗^
PF, deg	42.92 ± 4.34	41.38 ± 2.42	.116	45.10 ± 5.46	43.44 ± 3.59	.145	.125	.011^∗^
VAR, deg	20.92 ± 2.64	19.82 ± 3.32	.116	19.81 ± 3.30	17.81 ± 4.06	.096	.159	.043^∗^
VAL, deg	25.95 ± 3.35	24.29 ± 3.76	.153	24.82 ± 3.06	25.54 ± 3.21	.327	.191	.180

^a^Preoperative and postoperative values are showed as mean ± SD; AOFAS: American Orthopaedic Foot & Ankle Society score; KPAS: Karlsson-Peterson ankle score; CAIT: Cumberland Ankle Instability Tool score; VAS: Visual Analog Scale score; DF: dorsiflexion; PF: plantarflexion; VAR: varus; VAL: valgus. ^∗^The difference reached statistical significance (*P* < 0.05).

## Data Availability

All research data are available in the manuscript.
